# Targeting of vasoactive intestinal peptide receptor 2, VPAC2, a secretin family G-protein coupled receptor, to primary cilia

**DOI:** 10.1242/bio.20134747

**Published:** 2013-05-23

**Authors:** Livana Soetedjo, De'Vona A. Glover, Hua Jin

**Affiliations:** Department of Biological Sciences, University of Illinois at Chicago, Chicago, IL 60607, USA

**Keywords:** Primary cilia, VPAC2, VIPR2, Ciliary GPCR, Neuronal cilia, Glial cilia

## Abstract

Primary cilia protrude from the cell surface of many cell types in the human body and function as cellular antennae via ciliary membrane localized receptors. Neurons and glial cells in the brain possess primary cilia, and the malfunction of primary cilia may contribute to neurological deficits present in many cilia-associated disorders. Several rhodopsin family G-protein coupled receptors (GPCRs) are specifically localized to a subset of neuronal primary cilia. However, whether other family GPCRs target to neuronal cilia and whether glial primary cilia harbor any GPCRs are not known. We conducted a screening of GPCRs to determine their ability to target to primary cilia, and identified a secretin family member, Vasoactive Intestinal Receptor 2 (VPAC2), as a novel ciliary GPCR. Here, we show that endogenous VPAC2 targets to primary cilia in various brain regions, including the suprachiasmatic nuclei and the thalamus. Surprisingly, VPAC2 not only localizes to neuronal cilia but also to glial cilia. In addition, we show that VPAC2's C-terminus is both necessary and sufficient for its ciliary targeting and we define a novel ciliary targeting signal: the tetrapeptide RDYR motif in the C-terminus of VPAC2. Furthermore, we demonstrate that VPAC2 ciliary targeting is dependent on Tubby, the BBSome (a complex of Bardet–Biedl syndrome proteins) and the BBSome targeting factor, Arl6.

## Introduction

Primary cilia are typically solitary, immotile microtubule-based organelles present in many cell types in the mammalian body (Berbari et al., 2009). They harbor membrane receptors and their downstream targets, and therefore function as signaling hubs (Garcia-Gonzalo and Reiter, 2012; Nachury et al., 2010; Pazour and Bloodgood, 2008). Defects in the structure or function of primary cilia lead to ciliopathies with pleotropic phenotypes including cognitive impairment. The fact that clinical features of many ciliopathies include neurological deficits supports the notion that primary cilia play a role in brain function (Green and Mykytyn, 2010; Lee and Gleeson, 2011; Lee and Gleeson, 2010; Louvi and Grove, 2011). However, the lack of a complete catalog of ciliary components, especially membrane receptors, has impeded our understanding of signaling pathways mediated by cilia in the brain.

Most neurons in the brain possess a primary cilium (Bishop et al., 2007). A subset of neuronal cilia harbor certain G-protein coupled receptors (GPCRs) including somatostatin receptor 3 (SSTR3) (Händel et al., 1999), serotonin receptor 6 (5HT6) (Brailov et al., 2000; Hamon et al., 1999), melanin-concentrating hormone receptor 1 (MCHR1) (Berbari et al., 2008a; Berbari et al., 2008b), and dopamine receptor 1 (Domire et al., 2011). A recent study showed that GPR161, an orphan rhodopsin family GPCR, targets to neuronal cilia in primary hippocampal neuron culture (Mukhopadhyay et al., 2013). Interestingly, all ciliary GPCRs identified thus far belong to the rhodopsin family; whether GPCRs from other families target to neuronal primary cilia is not currently known.

Primary cilia in the brain are found in glia as well. Astrocytes (Bishop et al., 2007; Berbari et al., 2007; Yoshimura et al., 2011) and oligodendrocytes (Cenacchi et al., 1996; Louvi and Grove, 2011), but not microglia (Bishop et al., 2007; Sarkisian et al., 2013), have been shown to possess a primary cilium. Interestingly, SSTR3 proteins have so far only been detected in neuronal cilia (Berbari et al., 2007) and little is known regarding the expression and distribution of other ciliary GPCRs in glial cells (Sarkisian et al., 2013).

To expand the catalog of ciliary GPCRs in the brain, we performed an initial screening to identify GPCRs that can target to primary cilia in their GFP-tagged form and identified six GPCRs with this ability: Vasoactive Intestinal Peptide Receptor 2 (VPAC2, also known as VIPR2), Gastric Inhibitory Polypeptide Receptor (GIPR), G-protein coupled receptor 45 (GPR45), GPR63, GPR75 and GPR83.

We showed that endogenous VPAC2, a secretin family GPCR, localizes to primary cilia in various brain regions including the thalamus and the suprachiasmatic nuclei (SCN). VPAC2 plays important roles in the control of mammalian circadian rhythms in the SCN. Mice lacking VPAC2 show altered circadian rhythms in locomotor behavior, neuronal firing and clock gene expression (Aton et al., 2005; Cutler et al., 2003; Harmar et al., 2002; Maywood et al., 2006). Recent studies have also shown that duplication of the VPAC2 gene, and the resulting higher than normal VPAC2 signaling in patients confer a significant risk to schizophrenia (Beri et al., 2012; Levinson et al., 2011; Vacic et al., 2011).

We demonstrate that VPAC2 localizes to primary cilia not only in neurons but also in glial cells, including astrocytes and oligodendrocyte lineage cells. In addition, we showed that the C-terminus of VPAC2 is sufficient to target a non-ciliary membrane protein to cilia, and that a single amino acid mutation of the tetrapeptide RDYR in the C-terminus completely abolishes VPAC2 ciliary targeting. Furthermore, we show that the BBSome (a complex of Bardet–Biedl syndrome proteins), the BBSome targeting factor Arl6 and Tubby are important for ciliary targeting of endogenous VPAC2.

## Results

### Identification of novel ciliary GPCRs

To expand the catalog of ciliary GPCRs, we screened 122 non-olfactory GPCRs for their ability to target to primary cilia (for full list, see supplementary material Table S1). We transiently transfected GFP-tagged human or mouse GPCR constructs in mouse inner medullary collecting duct (IMCD3) cells and/or primary neuron cultures. Among those tested, we found two secretin family GPCRs (VPAC2 and GIPR) and four rhodopsin family orphan GPCRs (GPR45, GPR63, GPR75 and GPR83) that target to primary cilia (Fig. 1, Fig. 2A,B). Although known to couple with the same group of heterotrimeric G proteins, the secretin family GPCRs lack the classical signature sequences found in most members of the rhodopsin family GPCRs. By evaluating protein sequences, it has been proposed that the helical bundle of secretin family GPCRs is structurally distinct from that of rhodopsin family GPCRs (Foord et al., 2005; Fredriksson et al., 2003). Therefore, we suspected that VPAC2 and GIPR might have different ciliary targeting mechanisms compared to those of known ciliary GPCRs.

**Fig. 1.** Identification of novel ciliary GPCRs. GIPR-GFP, GPR45-GFP, GPR63-GFP, GPR75-GFP and GPR83-GFP target to primary cilia in IMCD3 cells. IMCD3 cells were transfected with plasmids expressing GIPR-GFP, GPR45-GFP, GPR63-GFP, GPR75-GFP or GPR83-GFP and serum starved to induce ciliogenesis. Cells were immunostained for acetylated α-tubulin (AcTubulin, red). DNA was labeled with mounting medium containing 4′,6-diamidino-2-phenylinodole (DAPI). Insets show unmerged images of the region around cilia. Scale bars: 5 µm.

**Fig. 2.** Endogenous VPAC2 localizes to primary cilia. (**A**,**B**) VPAC2-GFP and GFP-VPAC2 target to IMCD3 primary cilia. IMCD3 cells expressing VPAC2-GFP (A) or GFP-VPAC2 (B) were serum starved to induce ciliogenesis and immunostained for acetylated α-tubulin (AcTubulin, red). (**C**,**D**) Endogenous VPAC2 localizes to primary cilia in the thalamus and SCN regions of the rat brain. Rat thalamus (C) and SCN (D) cryosections were fixed and immunostained for VPAC2 (green) and Arl13B (red). Seventeen sections at 0.2 µm intervals were projected using sum over z-axis. (**E**) VPAC2 mRNA levels were reduced by ∼94% in thalamic cultures infected with lentivirus containing VPAC2 shRNAmiR #1 or VPAC2 shRNAmiR #2 compared to cells infected with control lentivirus. mRNA levels were measured by RT-qPCR. Error bars represent the standard deviation (SD) of triplicate PCR assays. ***P<0.001. GAPDH levels were used as an internal control for normalization. (**F**,**G**) VPAC2 localizes to primary cilia in thalamic neuron culture. Thalamic neuron culture was infected with lentivirus containing control shRNAmiR (F) or shRNAmiRs against VPAC2 (G) and immunostained for VPAC2 (green) and Arl13B (red). (**H**) Thalamic neuron culture cells were prepared and stained as in (F,G). Approximately 450 cilia were counted and the percentage of VPAC2 positive cilia was plotted. Error bars represent the SD among three different coverslips. (**I**,**J**) VPAC2 localizes to primary cilia in SCN neuron culture. SCN neuron culture was infected with lentivirus containing control shRNAmiR (I) or shRNAmiRs against VPAC2 (J) and immunostained for VPAC2 (green) and Arl13B (red). (**K**) SCN neuron culture cells were prepared and stained as in (I,J). Approximately 200 cilia were counted and the percentage of VPAC2 positive cilia was plotted. Error bars represent the SD among microscopic fields. (A–D,F,G,I,J) DNA was labeled with DAPI. Insets show unmerged images of the region around a cilium. Scale bars: 5 µm.

### Endogenous VPAC2 localizes to primary cilia in the brain

We first investigated whether endogenous VPAC2 and GIPR localize to primary cilia. We were unable to find an antibody against GIPR that could be validated in vivo, therefore we focused on VPAC2 and studied its ciliary trafficking exclusively. In the brain, VPAC2 is strongly expressed in several regions including the suprachiasmatic nuclei (SCN) and the thalamus (Sheward et al., 1995). We co-stained brain cryosections from 7-day-old rat pups with antibodies against VPAC2 and a ciliary marker, Arl13B (Caspary et al., 2007) and observed that the anti-VPAC2 antibody stained cilia in various brain regions including the thalamus and SCN (Fig. 2C,D). The anti-VPAC2 antibody also stained primary cilia in both thalamic and SCN neuron cultures (Fig. 2F,I). Cilium staining was lost when endogenous VPAC2 was depleted using lentivirus-mediated constructs that encode synthetic small hairpin RNA sequences within the context of a microRNA (shRNAmiR) (Fig. 2F–K). The efficiency of shRNAmiR-mediated VPAC2 knockdown was assessed using RT-qPCR (Fig. 2E). Both shRNAmiRs resulted in over a 94% knockdown of endogenous VPAC2 mRNA expression. Taken together, our results show that endogenous VPAC2 localizes to primary cilia in various brain regions and primary cultures.

### Endogenous VPAC2 localizes to primary cilia of neurons and glial cells

To determine whether VPAC2 targets to neuronal cilia, we co-stained primary thalamic culture with antibodies against VPAC2, Arl13B and a neuronal marker, MAP2. We found that 42% of MAP2 positive cells had primary cilia and 93% of those cilia contained VPAC2 (Fig. 3A). Although our thalamic neurons were cultured under serum-free conditions, a significant number of cells were negative for MAP2, indicating that non-neuronal cells were present in our culture. Interestingly, we detected VPAC2-containing cilia from some of the MAP2 negative cells (Fig. 3A), suggesting that VPAC2 targets to primary cilia in non-neuronal cells.

**Fig. 3.** Endogenous VPAC2 localizes to primary cilia of neurons and glial cells. (**A**) VPAC2 localizes to primary cilia in neuronal (MAP2+) and non-neuronal (MAP2−) cilia in primary thalamic culture. Primary thalamic culture (DIV9) was immunostained for VPAC2 (green), MAP2 (white) and Arl13B (red). (**B**) VPAC2 localizes to primary cilia of astrocytes (GFAP+) in primary thalamic culture. Primary thalamic culture (DIV9) was immunostained for VPAC2 (green), GFAP (white), and Alr13B (red). (**C**) VPAC2 localizes to primary cilia of astrocytes (Aldh1L1+/GFAP+) in primary thalamic culture. Primary thalamic culture (DIV9) was immunostained for VPAC2 (green), GFAP (white), and Arl13B (red). (**D**) VPAC2 localizes to primary cilia of astrocytes (Aldh1L1+) in vivo. Brain cryosections from 7-day-old rat pups were fixed and immunostained for VPAC2 (green) and Aldh1L1 (red). (**E**,**F**) VPAC2 localizes to primary cilia of oligodendrocytes (Sox10+ or NG2+) in primary thalamic culture. Primary thalamic culture (DIV7) was immunostained for VPAC2 (green), Sox10 (white) and Arl13B (red) in panel E and VPAC2 (green), NG2 (white) and Arl13B (red) in panel F. (**G**) Microglial cells labeled with Iba1 do not possess VPAC2-positive cilia in primary thalamic culture. Primary thalamic culture (DIV7) was immunostained for VPAC2 (green), Iba1 (white) and Arl13B (red). (A–G) DNA was labeled with DAPI. Scale bars: 5 µm.

To determine whether VPAC2 targets to primary cilia of glia, we stained cells with various glial cell markers. For astrocytes, we used antibodies against the “traditional” marker GFAP as well as Aldh1L1, a highly specific antigenic marker for astrocytes (Cahoy et al., 2008; Yang, Y. et al., 2011). For oligodendrocyte lineage cells, we used antibodies against Sox10, which is only expressed by oligodendrocyte progenitor cells and oligodendrocytes in the brain (Maka et al., 2005; Kang et al., 2010) and NG2, which is a marker for oligodendrocyte progenitor cells (Stallcup et al., 1990; Kang et al., 2010). For microglia, we used an antibody against Iba1, a microglia-specific calcium-binding protein (Imai et al., 1996).

Of the cells that were positive for GFAP (Fig. 3B) or for both GFAP and Aldh1L1 (Fig. 3C), approximately 53% of them possessed VPAC2-positive cilia. Furthermore, we detected VPAC2-positive cilia in Aldh1L1+ cells from brain cryosections of 7-day-old rat pups (Fig. 3D). Taken together, we concluded that VPAC2 targets to primary cilia of astrocytes in vivo and in vitro. Under our culture conditions, less than 1% of cells were Sox10 or NG2 positive, while ∼10% of those cells had primary cilia and 50% of those cilia were VPAC2-positive (Fig. 3E,F). We failed to detect any Arl13B-positive cilia in cells co-labeled with Iba1 (Fig. 3G), consistent with previous reports that microglia may not possess a primary cilium (Bishop et al., 2007; Sarkisian et al., 2013). Together, our results suggest that VPAC2 localizes to primary cilia in both neurons and glial cells such as astrocytes and oligodendrocyte lineage cells.

### The C-terminus is sufficient and necessary for VPAC2 ciliary targeting

As VPAC2 belongs to the secretin family, which does not share sequence homology with the rhodopsin family, we suspected that VPAC2 might have a different ciliary targeting mechanism compared to known rhodopsin family GPCRs. To study the ciliary targeting of VPAC2, we first tested two VPAC2 homologs for their ability to target to the primary cilium: Vasoactive Intestinal Peptide Receptor 1 (VPAC1, also known as VIPR1) and Pituitary Adenylate Cyclase-activating Polypeptide type 1 Receptor (PAC1, also known as ADCYAP1R1). Neither human VPAC1-GFP (hVPAC1-GFP) nor hPAC1-GFP targeted to IMCD3 primary cilia (Fig. 4A). Since most of the differences between VPAC2 and its homologs are concentrated in their C-terminal tails (supplementary material Fig. S1), we tested whether the C-terminus of VPAC2 is sufficient to target the non-ciliary membrane protein CD8α to cilia (Fig. 4B). CD8α is a well-characterized non-ciliary membrane protein that has been used in chimeras to identify ciliary targeting domains (Follit et al., 2010). As shown in Fig. 4D, a chimera protein CD8α-hVPAC2-Cterm-GFP containing the extracellular and transmembrane domains of CD8α and the C-terminus of VPAC2 targeted to primary cilia, while CD8α-GFP, CD8α-hVPAC1-Cterm-GFP, and CD8α-hPAC1-Cterm-GFP failed to do so (Fig. 4C,F,G). The hVPAC2-Cterm contains 58 amino acids with the last 44 amino acids differing significantly from those of VPAC1 and PAC1 (supplementary material Fig. S1). Interestingly, a chimera of CD8α-hVPAC2-Cterm44-GFP also targeted to primary cilia (Fig. 4E). Together, these results strongly suggest that the last 44 amino acids of VPAC2 are sufficient for ciliary targeting.

**Fig. 4.** The C-terminus is sufficient and necessary for VPAC2 ciliary targeting. (**A**) VPAC2-GFP (but not VPAC1-GFP and PAC1-GFP) targets to primary cilia in IMCD3 cells. IMCD3 cells were transduced with lentivirus vectors expressing VPAC2-GFP, VPAC1-GFP or PAC1-GFP and were serum starved to induce ciliogenesis. Cells were immunostained for acetylated α-tubulin (AcTubulin, red). (**B**) Schematic of CD8α chimeras. (**C–G**) The last 44 amino acids of VPAC2's C-terminus are sufficient to target the non-ciliary membrane protein CD8α to primary cilia. IMCD3 cells expressing GFP-tagged CD8α, CD8α-VPAC2-Cterm, CD8α-VPAC2-Cterm44, CD8α-PAC1-Cterm and CD8α-VPAC1-Cterm were serum starved and immunostained for AcTubulin (red). DNA was labeled with DAPI (C–G). Insets show an unmerged image of the region around the cilium. Scale bars: 5 µm.

### RDYR motif at the C-terminus is required for VPAC2 ciliary targeting

We next sought to determine which residues of VPAC2's C-terminus are required for VPAC2 ciliary targeting. This region does not contain a known ciliary targeting signal (CTS): an Ax[S/A]xQ motif identified in most neuronal ciliary GPCRs including SSTR3, 5HT6, MCHR1 and D1 (Berbari et al., 2008a; Domire et al., 2011), an [I/V]KARK motif found in GPR161, or a VxP motif that has been proposed to be a general CTS (Deretic et al., 2005; Geng et al., 2006). To identify the CTS of VPAC2, we conducted alanine-scanning mutagenesis of the last 44 amino acids of VPAC2, and tested their subcellular localization in IMCD3 cells. Most alanine mutations did not affect ciliary targeting of VPAC2, with the exception of the RDYR to ADAA mutation that completely abolished VPAC2 ciliary targeting (Fig. 5A; supplementary material Fig. S2). RDYR is a highly conserved tetrapeptide motif in VPAC2 proteins, from zebrafish to human (supplementary material Fig. S1). Interestingly, we found that single mutations in the RDYR motif resulted in the complete failure of VPAC2 targeting to cilia (supplementary material Fig. S3). We further confirmed these results in SCN neuron culture (Fig. 5B–G). Thus, the RDYR motif is necessary for ciliary targeting of VPAC2.

**Fig. 5.** The RDYR motif is necessary for VPAC2 ciliary targeting. (**A**) Summary of the alanine-scanning mutagenesis performed for the last 44 amino acids of the VPAC2 C-terminus. IMCD3 cells expressing GFP tagged VPAC2 harboring indicated alanine mutations (*GFP tag is in the N-terminus) were serum starved (supplementary material Fig. S2). The RDYR→ADAA mutation but not others abolished ciliary localization of GFP tagged VPAC2. (**B**) VPAC2-GFP localizes to primary cilia in SCN cells. SCN cells expressing VPAC2-GFP were immunostained for MAP2 (white) and Arl13B (red). (**C–G**) RDYR motif is required for VPAC2 ciliary targeting. SCN cells expressing VPAC2 harboring the RDYR→ADAA mutation or single mutations in the RDYR motif were immunostained for MAP2 (white) and Arl13B (red). DNA was labeled with DAPI (B–G). Insets show an unmerged image of the region around the cilium. Scale bars: 5 µm.

### The BBSome, Arl6 and Tubby are important for ciliary localization of VPAC2

Several proteins and protein complexes including the BBSome, the BBSome targeting factor Arl6 and Tubby have been shown to play key roles in neuronal cilia localization of endogenous SSTR3 and/or MCHR1 (Berbari et al., 2008b; Jin et al., 2010; Sun et al., 2012). To test whether the same targeting machinery is used by VPAC2, we depleted BBS2 (a BBSome subunit), Arl6 and Tubby by lentivirus-mediated RNAi in thalamic neuron culture. BBS2 and Tubby shRNAmiRs showed more than a 93% reduction in mRNA levels (Fig. 6A,B). To knockdown Arl6 in neuronal cultures, we used mArl6shRNAs, which have been shown to effectively knockdown Arl6 in mouse neuronal cells (Jin et al., 2010), and confirmed that they lowered the Arl6 protein level (Fig. 6C). As shown in Fig. 6D–G, knocking down Arl6, BBS2 or Tubby abolished ciliary targeting of VPAC2. Thus, Tubby and the BBSome/Arl6 are important for ciliary targeting of endogenous VPAC2.

**Fig. 6.** The BBSome, Arl6 and Tubby are required for VPAC2 ciliary targeting. (**A**,**B**) BBS2 and Tubby mRNA levels were reduced by more than 93% in rat thalamic cultures infected with lentivirus containing shRNAmiR against BBS2 (A) or Tubby (B) compared to cells infected with control lentivirus. mRNA levels were measured by RT-qPCR. Error bars represent the SD of triplicate PCR assays. ***P<0.001. GAPDH levels were used as an internal control for normalization. (**C**) Protein extracts from mouse thalamic cultures infected with control shRNA or Arl6 shRNAs were immunoblotted for Arl6 and actin (loading control). (**D**) Tubby and BBS2 are required for VPAC2 ciliary targeting. Rat thalamic cells were infected with lentivirus containing control shRNAmiR and shRNAmiRs against Tubby or BBS2 and immunostained for VPAC2 (green) and Arl13B (red). (**E**) Thalamic neuron culture cells were prepared and stained as in panel D. Approximately 500 cilia were counted and the percentage of VPAC2 positive cilia was plotted. (**F**) Knockdown of Arl6 affects VPAC2 ciliary targeting. Thalamic cultures were infected with control shRNA or Arl6 shRNAs or immunostained for VPAC2 (green) and Arl13B (red). (**G**) Arl6 is required for VPAC2 ciliary targeting. Rat thalamic neuron culture cells were prepared and stained as in panel F. Approximately 600 cilia were counted and the percentage of VPAC2 positive cilia was plotted. Error bars represent the SD among three different coverslips (E,G). ***P<0.001. DNA was labeled with DAPI <2?show=[to]?>(D,F). Insets show unmerged images of the region around a cilium highlighted with a white arrow. Scale bars: 5 µm.

## Discussion

We expanded the catalog of ciliary GPCRs and demonstrated for the first time that a secretin family GPCR, VPAC2, localizes to primary cilia not only in neurons but also in glial cells including astrocytes and oligodendrocytes (Fig. 3), thereby implicating the involvement of both neuronal and glial primary cilia in VPAC2-mediated signaling. We showed that VPAC2 localizes to primary cilia in various brain regions including the SCN and the thalamus (Fig. 2). The fact that VPAC2 localizes to cilia in the SCN implies that ciliary VPAC2 signaling may play a role in regulating circadian rhythm. Although there has been no prior investigation of a circadian rhythm phenotype in BBS or Tubby mutant mice or mice lacking cilia in the brain, many ciliary defect-associated pathological conditions such as obesity, hypertension and psychotic conditions are associated with abnormalities in circadian rhythms. The fact that VPAC2 localizes to cilia in various brain regions suggests that abnormal ciliary VPAC2 signaling may contribute to schizophrenia in patients with a gene duplication of VPAC2. This is in line with recent findings suggesting psychiatric diseases such as schizophrenia may result from defects in primary cilia-dependent signaling (Doherty, 2009; Marley and von Zastrow, 2010; Marley and von Zastrow, 2012).

Unlike SSTR3, 5HT6 and MCHR1, the C-terminus of VPAC2 is sufficient to target a non-ciliary membrane protein, CD8α, to primary cilia (Fig. 4). We further identified a novel ciliary targeting signal, the tetrapeptide RDYR motif in the C-terminus of VPAC2, and showed that single amino acid mutations in this motif abolish ciliary targeting (Fig. 5). Interestingly, although VPAC2 belongs to the secretin family, and contains a different CTS compared to that of SSTR3 and MCHR1, VPAC2 ciliary targeting is dependent on the same set of proteins including the BBSome, Arl6 and Tubby (Fig. 6). As Bardet–Biedl syndrome (BBS), is most likely the result of ciliary protein targeting failure (Jin et al., 2010), the failure to traffic VPAC2 to cilia might contribute to the pleiotropic phenotype exhibited by BBS patients. Whether ciliary targeting of other GPCRs (GIPR, GPR45, GPR63, GPR75 and GPR83) is also dependent on the BBSome, Arl6 or Tubby remains unknown, and requires further investigation.

As VPAC2-mediated signaling may be important for maintaining circadian rhythms and normal brain function, our research on VPAC2 ciliary trafficking provides a new avenue for future investigations into the role of ciliary VPAC2 signaling in the control of circadian rhythms and in psychotic diseases such as schizophrenia.

## Materials and Methods

### Animals

Mice and rats were purchased from Charles Rivers (Wilmington, MA, USA). Animal care and use was in accordance with the National Institutes of Health Guide for the Care and Use of Laboratory Animals, and was approved by the Institutional Laboratory Animal Care and Use Committee at the University of Illinois at Chicago.

### Plasmids

Human VPAC2 and PAC1 ORFs (BC010569, BC117116) were obtained from the human ORFeome collection (Open Biosystems, Waltham, MA, USA). VPAC1 (BC064424) was obtained from the human ORFeome v8.1 collection (Yang, X. et al., 2011). The CD8α chimeras were generated by replacing CD8α C-terminal amino acids (aa) 213–235 with the C-termini of VPAC2 (aa 380–438), VPAC1 (aa 394–457), PAC1 (aa 406–468) and the partial C-terminus of VPAC2 (aa 395–438) (for primers used to construct CD8α chimeras, please refer to supplementary material Table S2). VPAC2 alanine scanning mutants were generated with Phusion DNA Polymerase. All constructs for transient transfection were subcloned into pEF5α.FRT derivatives and all lentivirus expression constructs were subcloned into a pCDH.EF1 derivative (System Biosciences, Mountain View, CA, USA). DNA constructs were confirmed by restriction digestion and sequencing (RRC-DNAS, Chicago, IL, USA).

### Cell culture

IMCD3 and 293FT cells were maintained in DMEM:F12 (IMCD3) or DMEM high glucose (293FT) supplemented with 10% Fetal Bovine Serum, 100 units per ml penicillin and 100 µg/ml streptomycin at 37°C and 5% CO_2_. Plasmid transfections in IMCD3 cells were performed with Lipofectamine 2000 (Life Technologies, Grand Island, NY, USA). IMCD3 cells were serum starved in DMEM:F12 and supplemented with 0.2% Fetal Bovine Serum, 100 units per ml penicillin and 100 µg/ml streptomycin, 16–24 hours after transfection to induce ciliogenesis. Cells were examined between 40–48 hours post transfection.

For SCN cultures, P1–P5 rat (Sprague Dawley) pups were decapitated, their brains dissected and placed in Hank's Balanced Salt Solution (Sigma, St. Louis, MO, USA). Three hundred µm coronal sections were cut using a tissue slicer from Stoelting (Wood Dale, IL, USA). Under a dissection microscope, the sections containing the mid-part of the SCN were selected and the SCN region was cut out using a scalpel. Cells were enzymatically digested with papain (Worthington, Lakewood, NJ, USA) for 45 min at 37°C. Cells were then triturated and 20 µl of the cell suspension containing 5×10^4^ cells were placed over coverslips (12 mm diameter) coated with PDL and Laminin (BD Biosciences, San Jose, CA, USA). One ml of NBactiv4 (BrainBits, Springfield, IL, USA) was added after 30 min. The medium was changed once every two to three days. Cells were transfected with Lipofectamine 2000 on days in vitro 5 (DIV5) and examined on DIV7.

For thalamic cultures, P1 mouse or rat pups (CD-1 mouse or Sprague Dawley rat) were decapitated and their thalami were dissected. Cells were enzymatically digested with papain for 45 min at 37°C. Cells were then triturated and 20 µl cell suspension containing 2×10^4^ cells were placed over the coverslip (12 mm diameter) coated with PDL (Sigma P7405). One ml of NBactiv4 was added after 30 min. The medium was changed once every four to five days. Cells were transfected with Lipofectamine 2000 on DIV5 and examined on DIV7.

### Cryosection

P7 rats (Wistar rat) were decapitated and their brains were dissected, then washed in phosphate buffered saline (PBS) briefly, and immersed in 4% paraformaldehyde at 4°C overnight. Fixed specimens were then immersed in 15% sucrose (w/v) diluted in PBS for 48 hours and 30% sucrose (w/v) for 24 hours. All tissues were placed in Tissue Tek OCT (Sakura Finetek, Torrance, CA) and frozen over liquid nitrogen. Seven µm coronal sections were cut at −20°C using a Vacutome Cryostat (Microm International GmbH, Waldorf, Germany) and collected on 3-Aminopropyltriethoxysilane coated slides.

### Immunofluorescence and microscopy

IMCD3, SCN and thalamic cells were fixed in 4% paraformaldehyde in PBS for 10 min at room temperature. Cells were then blocked with 5% normal donkey serum for IMCD3 cells (2% for neuron cultures) in buffer containing 0.1% Triton X-100 for 40 min at room temperature. Primary antibodies were then applied for one hour at room temperature, and secondary antibodies (Alexa Fluor 488, 546 or 647, Life Technologies) were applied for 30 min at room temperature. Coverslips were then mounted using Vectashield containing 4′,6-diamidino-2-phenylindole (DAPI) (Vector Laboratories, Burlingame, CA, USA). Cryosections were fixed with 4% paraformaldehyde in PBS for 10 min at 4°C. Sections were then blocked with 5% normal donkey serum in PBST (PBS with 0.2% Tween-20) for 40 min. Primary antibodies were then applied overnight at 4°C, and secondary antibodies were applied for 30 min at room temperature. Nuclei were stained with Vectashield containing DAPI (Vector Laboratories). Images were acquired on Delta Vision Elite (GE, Schenectady, NY, USA). Forty to fifty sections at 0.2 µm intervals were acquired using 60× oil NA 1.4 objective and the section containing cilia was selected for each figure panel unless described otherwise.

### shRNAmiR lentivirus production and knockdown

shRNAmiR lentivirus constructs were prepared according to Allaire et al. (Allaire et al., 2010) with slight modifications. Target sequences for ratVPAC2, ratBBS2 and ratTubby were designed using the Block-iT RNAi Designer (Life Technologies, Carlsbad, CA, USA) and subcloned into pCDNA6.2/GW-EmGFP-miR (Life Technologies) to obtain the shRNAmiR knockdown constructs. The EmGFP-shRNAmiR cassette was then amplified by the polymerase chain reaction (PCR) and subcloned into a pCDH.EF1 derivative (For primers used in this experiment, please refer to supplementary material Table S3).

For virus production, 293FT cells were co-transfected with the pCDH vector, pSPAX2 (packaging vector) and pMD2.G (envelope vector) using Polyethylenimine Max (Polysciences, Warrington, PA, USA). The medium was changed after 16–20 hours, and the supernatant was collected and filtered (0.45 µm) after 48–72 hours. The virus was then concentrated with PEG-it (System Biosciences). The precipitated lentivirus was suspended with cold PBS, aliquot and stored at −80°C until use.

Thalamic cultures and SCN cultures were infected with lentivirus harboring shRNAmiRs on either DIV1 or DIV2. Immunostaining was conducted on DIV7.

### RNA isolation, cDNA synthesis and real time quantitative PCR (RT-qPCR)

Cultured thalamic neurons were lysed and total RNA was extracted using RNeasy Mini Kit (Qiagen, Valencia, CA, USA). The QuantiTect Reverse Transcription Kit (Qiagen) was used to reverse transcribe the mRNA into complementary DNA (cDNA). Real-time quantitative PCR was performed to amplify VPAC2, BBS2 and Tubby with specific primer sets (refer to supplementary material Table S4 for primer sequences). The template (5 ng) was amplified in 20 µl reaction volumes using SYBR Green PCR Master Mix (Applied Biosystems, Foster City, CA, USA). Data collection was performed on the ABI ViiA 7 and normalized to GAPDH. Each sample was assayed in triplicate. The relative standard curve method was used for analyzing quantitative PCR (qPCR) data.

### Antibodies and dilutions

The commercial antibodies used were against: VPAC2 (Rabbit, 1:100, ab28624, Abcam, Cambridge, MA, USA), actin (Rabbit, 1:1000, A2066, Sigma), Arl13B (Mouse, 1:2000, 75–287, UC Davis/NIH NeuroMab Facility, Davis, CA, USA), Aldh1L1 (Mouse, 1:1000, 75-164, UC Davis/NIH NeuroMab Facility), acetylated α-tubulin (Mouse, 1:5000, mAb 6-11B-1, Sigma), GFAP (Chicken, 1:5000, ab4674, Abcam), MAP2 (Chicken, 1:5000, ab92434, Abcam) and Iba1 (Goat, 1:500, ab5076, Abcam). Antibodies against Sox10 (Guinea pig, 1:1000), NG2 (Guinea pig, 1:1000) and Arl6 (Rabbit, 1:1000) were gifts from Drs Wegner, Stallcup and Nachury, respectively.

## Supplementary Material

Supplementary Material
